# Evidence-Based Analysis of the Emergency Temporary Cardiac Pacing (Electrical Stimulation from Metal Wire Electrode)

This article has been retracted.

**DOI:** 10.1155/2021/5677598

**Published:** 2021-08-25

**Authors:** Meng Liu, Xuming Lin, Qiaoyin Tan, Xiaotong Han

**Affiliations:** ^1^Emergency Department, Hunan Provincial People's Hospital (The First-Affiliated Hospital of Hunan Normal University), Changsha 410005, Hunan, China; ^2^Electromyogram Department, Hunan Province Hospital of Chinese Medicine (The Second-Affiliate Hospital of Hunan University of Chiniese Medicine), Changsha 410005, China; ^3^College of Teacher Education, Zhejiang Normal University, Jinhua 321004, Zhejiang, China

## Abstract

The patient's Cr (creatinine), BUN (blood urea nitrogen), HBG (hemoglobin), VT (ventricular tachycardia), pacing frequency, puncture point, emergency to permanent pacing time, pacing current (mA), pacing threshold current (mA), and admission diagnosis data were collected. The data were subjected to frequency statistics, curve regression analysis, PLS regression analysis, adjustment analysis, chi-square test, ridge regression analysis, discriminant analysis, negative binomial regression analysis, Poisson regression analysis, and stepwise regression analysis. Some findings include the following: (1) Cr has a significant positive effect on HBG, and BUN has a significant negative effect on HBG. (2) VT has a negative correlation with age and a positive correlation with CK-MB and CK (creatinine kinase). (3) Myocarditis has a negative correlation with age and a significant positive correlation with CTnI (cardiac troponin I). (4) AST (aspartate transaminase) and ALT (alanine aminotransferase) have a significant positive impact on DDI (D-dimer), while CTnI has a significant negative impact on DDI. MYO (myoglobin) has no impact relationship to DDI. (5) ALT has a significant positive relationship with APTT (partial thromboplastin time). (6) Alb (albumin) and TBIL (total bilirubin) have a significant positive effect on PLT (platelet) count, while pro-BNP (B-type natriuretic peptide) and MYO have a significant negative effect on PLT. (7) CK has a significant positive effect on INR (international normalized ratio). (8) The relationship between sinus node dysfunction and VT significantly affect the pacing frequency (beats/minute). For third-degree atrioventricular block, different samples of sinus node dysfunction showed significant differences. (9) There is a significant positive correlation between pacing current (mA) and pacing threshold current (mA). (10) There was a significant positive correlation between perceived voltage (mV) and the time from emergency to permanent pacing. Admission diagnosis has a significant positive impact on the time from emergency to permanent pacing. The change (increase) in time from emergency to permanent pacing was 1.137-fold when an additional condition was diagnosed on admission.

## 1. Introduction

As an implantable electronic therapeutic instrument, temporary transvenous cardiac pacing (TTCP) [1] is widely used in life-threatening slow arrhythmia, hemodynamic damage, and transient bradycardia caused by the underlying pathology of patients. The standard TTCP pacing lead [2, 3] has no fixed mechanism and has a blunt and smooth hard tip. The negative electrode of the lead is in direct contact with the myocardium to conduct electrical stimulation [4]. Therefore, the tip of the negative electrode of the lead has a potential risk of penetrating the myocardium in the clinical application of TTCP, which leads to serious complications of cardiac perforation. The incidence of sudden cardiac death in patients can be high around 1/3 if other operations are also underway [5].

The key of temporary cardiac pacing device placement is electrode placement. Implantation of electrode tip into the apex of right ventricle is the best position for stable pacing and difficult dislocation. Electrode implantation can usually be performed under fluoroscopy [6, 7], but this operation technique is highly professional and fluoroscopy will expose patients to radiation. Ultrasonic guidance is also an optional scheme, but it requires higher ultrasonic technology [8]. Pacing capture from surface electrocardiogram (ECG) monitoring is a common bedside technique [9], also known as blind insertion, which easily leads to atrial perforation, and the probability of implantation in the best position (right ventricular apex) is only 44%. Blind insertion (ECG monitoring on body surface) and implantation under X-ray cannot judge the degree of contact between the electrode tip and electrode [10, 11]. Using these two methods, it is not uncommon for electrodes to insert into the myocardium and penetrate through the atrial or ventricular wall in severe cases.

The technical factors are important for the success of a TTCP operation. From another angle, the patient characteristics are also important for a TTCP operation. However, this angle has been rarely studied based on clinical cases. Evidence-based analysis plays a key role in understanding clinical observations [12, 13]. This work presents an evidence-based analysis of the emergency temporary cardiac pacing (electrical stimulation from metal wire electrode) for the reasons of severe bradycardia or tachycardia. The findings may be used alongside the technical factors, leading to better TTCP operations.

## 2. Objective and Methods

The retrospective study involves consecutive 21 patients who had intracavity ECG-guided TTCP at the emergency department of Hunan Provincial People's Hospital from November 2018 to October 2020. One case was excluded as electrodes were placed in the right atrium for atrial overspeed inhibition. Eligible 20 cases' electrodes were placed in the right ventricle, requiring emergency temporary cardiac pacing due to severe arrhythmia (Table 1). From the perspective of gender, there are relatively more “males” in the sample. The indication of TTCP include sinus node dysfunction (SND) was 6, atrioventricular block (AVB) was 16, ventricle tachycardia (VT) was 4. 19 patients had severe symptoms, either with syncope (16) or after CPR (3). The age was in the range of 64.55 ± 8.75. The collected raw data is shown in Supplementary Materials. The information is analyzed using SPSS. Some cases may be excluded if the information of some patients is not available for a SPSS analysis.

## 3. Results and Discussion

It can be seen from Table 2 that using Cr and BUN as independent variables and HBG as a dependent variable for Poisson regression analysis, it can be seen from Table 2 that the model pseudo-R formula (McFadden's R formula) is 0.100, which means that Cr and BUN can explain the reason for the 10.0% change of HBG. From the above table, the model equation is log (*U*) = 4.822 + 0.002*∗*Cr − 0.034*∗*BUN (where *U* represents the expected mean).

According to the analysis, Cr has a significant positive effect on HBG. And, a dominance ratio (OR value) of 1.002 means that when Cr is increased by one unit, the magnitude of the change (increase) in HBG is 1.002-fold.

The regression coefficient value of BUN was −0.034, and it showed a significant difference at 0.01 level (*Z* = −4.573, *p* < 0.01), indicating that BUN had a significant negative effect on HBG. And, an OR of 0.966 meant that there was a 0.966-fold change in HBG when BUN was increased by one unit.

According to the summary analysis, Cr in total has a significant positive effect on HBG, and BUN in total has a significant negative effect on HBG.

As shown in Table 3, correlation analysis was performed to determine the correlation between locomotor speed and age, CK-MB, and CK, and Pearson correlation coefficient was used to indicate the strength of the correlation. Specific analysis shows the following.

The coefficient for VT and age was −0.481, showing a significant difference of 0.05, thus indicating a significant negative correlation between VT and age. The correlation coefficient between VT and CK-MB is 0.458, and it shows the significance of 0.05 level, thus indicating that there is a significant positive correlation between VT and CK-MB. The correlation coefficient between VT and CK is 0.523, and it shows the significance of 0.05 level, thus indicating that there is a significant positive correlation between VT and CK.

In conclusion, there is a significant negative correlation between VT and age and a significant positive correlation between VT and CK-MB and CK.

As shown in Table 4, correlation analysis was used to study the correlation between myocarditis and age, CTnI, and Pearson correlation coefficient was used to indicate the strength of the correlation. Specific analysis shows the following.

The correlation coefficient between myocarditis and age was −0.669 and showed a significance of 0.01, thus indicating a significant negative correlation between myocarditis and age. The correlation coefficient between myocarditis and CTnI is 0.838, and it shows the significance of 0.01 level, thus indicating that there is a significant positive correlation between myocarditis and CTnI.

Table 5 shows the summary of 5 Poisson regression analysis results (*n* = 19). From the table, we can see that the pseudo-R formula of the model (McFadden's R formula) is 0.737, meaning that AST, ALT, MYO, and CTnI induce 73.7% change of DDI. As shown in Table 5, the model equation is log (*U*) = 0.101 + 0.014*∗*AST + 0.004*∗*ALT−0.003*∗*MYO-0.553*∗*CTnI (where *U* represents the expected mean).

According to the analysis, the regression coefficient of AST was 0.014, showing a significant relationship of 0.01 (*z* = 4.093, *p* < 0.001), indicating that AST had a significant positive effect on DDI. And, a dominance ratio (OR value) of 1.014 means that a unit increase in AST results in a 1.014-fold increase in DDI.

The regression coefficient of ALT was 0.004 and was significant at 0.01 (*z* = 3.506, *p* < 0.001), indicating a significant positive effect of ALT on DDI. And, an odds ratio (OR value) of 1.004 means that when ALT was increased by one unit, the magnitude of the change (increase) in DDI was 1.004-fold.

The regression coefficient for MYO was −0.003, but it was not significant (*z* = −1.944, *p*=0.052 >0.05), suggesting that MYO had no effect on DDI.

The coefficient of CTnI was −0.553, which significantly indicated that CTnI had a significant negative effect on DDI. Summary analysis showed that AST and ALT had a significant positive impact on DDI, and CTnI had a significant negative impact on DDI. However, MYO does not have an impact relationship with DDI.

Curve regression is a regression analysis method for variables with nonlinear relationship. Curve regression is a nonlinear relationship in relation form, but it can be changed into a linear relationship through various conversions, and finally, the regression model is established. As shown in Table 6, *p*=0.044, less than 0.05 showed a significant relationship, indicating that the independent variable ALB had an influence on the dependent variable HBG. Specifically shown in Figure 1, namely, the ALB and HBG quadratic curve fitting:

As shown in Table 7, Poisson regression analysis was performed using pro-BNP, MYO, ALB, and TBIL as independent variables and PLT as the dependent variable. From Table 7, it can be seen that the model pseudo-R square (McFadden's R square) was 0.603, meaning that pro-BNP, MYO, ALB, and TBIL could explain the change reason of PLT by 60.3%. As shown in Table 7, the model equation is log (*U*) = 4.152−0.000*∗*Pro-BNP−0.000*∗*MYO + 0.027*∗*ALB + 0.004*∗*TBIL (where *U* represents the expected mean). The regression coefficient of pro-BNP was −0.000, and the value was noticeable at 0.01 level (*z* = −6.033, *p* < 0.001), indicating that pro-BNP had a significant negative effect on PLT. And, an OR of 1.000 meant that there was a 1.000-fold change in PLT when pro-BNP was increased by one unit.

The regression coefficient value of MYO was 0, and it was significant at 0.01 level (*z* = −3.917, *p* < 0.001), indicating that MYO had a significant negative effect on PLT. And, the odds ratio (OR value) was 1.000, meaning that when MYO was increased by one unit, the magnitude of the change (decrease) in PLT was 1.000-fold.

The regression coefficient value of ALB was 0.027, and it was significant at 0.01 level (*z* = 6.991, *p* < 0.001), which meant that ALB had a significant positive effect on PLT. And, a dominance ratio (OR value) of 1.028 means that there was a 1.028-fold increase in PLT when ALB was increased by one unit.

The regression coefficient of TBIL was 0.004 and was significant at 0.01 (*z* = 11.708, *p* < 0.001), indicating a significant positive effect of TBIL on PLT. And, a dominance ratio (OR value) of 1.004 means that the magnitude of the change (increase) in PLT was 1.004-fold when TBIL was increased by one unit.

According to the summary analysis, ALB ALB, and TBIL together have a significant positive impact on PLT, and pro-BNP and MYO together have a significant negative impact on PLT.

The stepwise regression model automatically identifies significant independent variable (*x*), and non-significant *x* is automatically removed from the model. CTnI, CK-MB, CK, ALB, AST and ALT were taken as independent variables, and APTT was taken as dependent variable for stepwise regression analysis. After automatic recognition by the model, finally, a total of 1 item of ALT was left in the model, as shown in Table 8. The model equation was APTT = 26.524 + 0.024*∗*ALT, and the R-square value was 0.516, meaning ALT could account for the 51.6% change in APTT. Moreover, the model passed the F-test (*F* = 18.150, *p* < 0.001 <0.05), indicating that the model was effective. In addition, the multicollinearity of the model is tested, and it is found that all the VIF values in the model are less than 5, which means that there is no collinearity problem. And the value of D-W is near the number 2, which indicates that the model has no autocorrelation and there is no correlation between the sample data, so the model is good. The regression coefficient of ALT was 0.024(*t* = 4.260, *p* < 0.001 <0.01), indicating a significant positive effect of ALT on APTT.

PLS regression is used to study the impact relationship of multiple X's on multiple Y's. PLS regression is generally used for regression research with small sample size and possible collinearity problem. The number of principal components was paired, and it usually needed to be judged by combining cross-validation with VIF index.  Table 9 shows the regression relationship expression between dependent variable *y* and independent variable *x*, including the relationship expression between each dependent variable *y* and all independent variables:

(1) $$\begin{array}{c} \text{RBC}=-0.126*\text{BUN}+0218*\text{AST}-0.602*\text{ALT}+0.678*\text{ALB}+0.011*\text{MYO}+0.424*\text{CTnI}, \end{array}$$

(2) $$\begin{array}{c} \text{WBC}=0.300*\text{BUN}+0.833*\text{AST}+0.005*\text{ALT}+0.310*\text{ALB}-0.110*\text{MYO}+0.079*\text{CTnI.} \end{array}$$

As shown in Table 10, CK-MB, CK, ALB, AST, ALT, pro-BNP were taken as independent variables, and INR was taken as dependent variable for stepwise regression analysis. After automatic recognition by the model, finally there was one remaining item of CK in the model. The model formula was as follows: INR = 0.906 + 0.000*∗*CK, and the R-square value was 0.592, which meant that CK could explain the 59.2% change in INR. Moreover, the model passed the F-test (*F* = 24.625, *p* < 0.001), indicating that the model was effective.

In addition, the multicollinearity of the model is tested, and it is found that all the VIF values in the model are less than 5, which means that there is no collinearity problem. And the value of D-W is near the number 2, which indicates that the model has no autocorrelation and there is no correlation between the sample data, so the model is good. The analysis shows that the regression coefficient of CK is 0.000(*t* = 4.962, *p* < 0.001), which means that CK has a significant positive effect on INR.

Table 11 shows that in this study, the treatment methods of independent variable (sinus node dysfunction) and regulatory variable (VT) were: centralized, and the dependent variable (pacing frequency (times/minute)) was not treated. The regulatory effects were divided into three models, with the independent variable (sinus node dysfunction) included in Model 1. In Model 2, the moderator variable (VT) was added on the basis of Model 1, and in Model 3, the interaction term (the product term of independent variable and moderator variable) was added on the basis of Model 2.

For Model 1, its purpose is to study the effect of independent variable (sinus node dysfunction) on dependent variable (pacing frequency (beats/min)) without considering the interference of regulatory variable (VT). As shown in Table 11, the independent variable (sinus node dysfunction) showed a significant difference (*t* = −2.271, *p* = 0.036 <0.05). This means that the sinus node dysfunction has a significant impact on the pacing frequency (beats/minute).

Looking at the significance of the interaction item in Model 3, it can be seen from Table 11 that the interaction item between sinus node dysfunction and VT did not show significance (*t* = 0.190, *p* = 0.852 >0.05). As well as model 1, it can be seen that when the adjustment variable (VT) is at different levels, the impact amplitude of sinus node dysfunction on pacing frequency (beats/min) is consistent.

As shown in Table 12, the independent variables that were exchanged between Model 1 and Model 2 were (VT) and the regulatory variable (sinus node dysfunction). For Model 1, its purpose is to study the effect of independent variable (VT) on dependent variable (pacing frequency (beats/min)) without considering the interference of regulatory variable (sinus node dysfunction). As shown in Table 12, the independent variable (VT) showed significant (*t* = −2.443, *p* = 0.025 <0.05). It means that VT has a significant influence on pacing frequency (beats/min).

As shown in Table 13, the chi-square test (cross-analysis) was used to study the independence of sinus node dysfunction for the third-degree atrioventricular block. From the above table, it can be seen that different samples of sinus node dysfunction showed significant effects on third-degree atrioventricular block (*p* < 0.05).

A research algorithm is used by ridge regression to solve the collinearity of independent variables in linear regression analysis. As shown in Figure 2 (ridge trace map), ridge regression makes the regression coefficient estimable by introducing *k* unit matrices. The introduction of unit array will lead to information loss, but at the same time, it can be exchanged with a reasonable estimate of the regression model. Ridge trace was obtained after ridge regression analysis using ventricular velocity, sinus node dysfunction, third-degree atrioventricular block, syncope/CPR, myocarditis, and acute myocardial infarction as independent variables and pacing frequency (times/min) as dependent variable. It can be seen that the normalized regression coefficient of the independent variable tends to be stable when the *k* value is 0.99.

As shown in Table 14, myocarditis has been known to have a significant relationship with the puncture point, and discriminant analysis was performed for both. A total of 20 data were studied in this discriminant analysis (LDA), and the first 90.00% of the data were selected as the training set to train the fitting discriminant analysis model. The remaining 10.00% was used as the test set to validate the model.

After the discriminant analysis, the accuracy of data prediction in the training set can be viewed and judged by three indicators, namely, accuracy rate, recall rate, and *F*1 score. First, the accuracy rate refers to the proportion of samples belonging to category 2 (within the right neck) when the model predicts this category. Second, the recall rate refers to the proportion of samples correctly predicted for category 2 (within the right neck) when it is actual. Finally, the *F*1 score value refers to the weighted comprehensive index of correct rate and recall rate, and its calculation formula is *F*1 score = 2*∗*correct rate*∗*recall rate/(correct rate + recall rate). The values of these three indexes are all greater than 60%, indicating that the statistical puncture point of myocarditis is in the right neck when the sample size is 22.

As shown in Table 15, correlation analysis was used to study the correlation between perceived voltage (mV), pacing current (mA), and the total of two items, namely, emergency to permanent pacing time and pacing threshold current (mA). Pearson correlation coefficient was used to indicate the strength of the correlation.

The specific analysis shows that the correlation coefficient between perceived voltage (mV) and emergency to permanent pacing time is 0.746, and it shows the significance of 0.05 level, thus indicating that there is a significant positive correlation between perceived voltage (mV) and emergency to permanent pacing time. The correlation coefficient value between pacing current (mA) and pacing threshold current (mA) is 0.719, and it shows the significance of 0.01 level, thus indicating that there is a significant positive correlation between pacing current (mA) and pacing threshold current (mA).

As shown in Table 16, a total of 1 item of admission diagnosis was taken as the independent variable, and the negative binomial regression analysis was performed with the emergency to permanent pacing time as the dependent variable. From the above table, it can be seen that the model formula was as follows: log(*Y*) = 2.373 + 0.128*∗*admission diagnosis. The regression coefficient of admission diagnosis was 0.128, and the significance was shown at 0.05 level (*z* = 2.401, *p*=0.016 <0.05), which meant that the admission diagnosis had a significant positive impact on the time from emergency to permanent pacing. And, an odds ratio (OR value) of 1.137, which means that the change from emergency to permanent pacing time was 1.137-fold when an additional condition was diagnosed on admission. Summary analysis shows that admission diagnosis will have a significant positive impact on the time from emergency to permanent pacing.

The above studies have found that mathematical analysis is conducive to understand the patients' conditions of emergency temporary cardiac pacing and clarify the relationship between various physical indicators. Such an analysis was used to establish a biological model of the heart block in the study of Cingolani et al. [14] and real-time tracking of intrathoracic impedance sensors in the study of DeArmond et al. [15]. Similarly, Carson and Tseng [16] performed regression analysis on various indicators of ECG of patients. These studies have highlighted the advantages of mathematical analysis in medical research to better display the research results and conclusions.

## 4. Conclusions

Data analysis was performed on 20 patients. The patient's Cr, BUN, HBG, VT, pacing frequency, puncture point, emergency to permanent pacing time, pacing current (mA), pacing threshold current (mA), and admission diagnosis data were collected. The data were subjected to frequency statistics, curve regression analysis, PLS regression analysis, adjustment analysis, chi-square test, ridge regression analysis, discriminant analysis, negative binomial regression analysis, Poisson regression analysis, and stepwise regression analysis. Some findings include the following: Cr has a significant positive effect on HBG, and BUN has a significant negative effect on HBG. VT has a negative correlation with age and a positive correlation with CK-MB and CK. Myocarditis has a negative correlation with age and a significant positive correlation with CTnI. AST and ALT have a significant positive impact on DDI, while CTnI has a significant negative impact on DDI. MYO has no impact relationship to DDI. ALT has a significant positive relationship with APTT. ALB and TBIL have a significant positive effect on PLT, while pro-BNP and MYO have a significant negative effect on PLT. CK has a significant positive effect on INR. The relationship between sinus node dysfunction and VT significantly affecting the pacing frequency (beats/minute). For the third-degree atrioventricular block, different samples of sinus node dysfunction showed significant differences. There was a significant positive correlation between pacing current (mA) and pacing threshold current (mA). There was a significant positive correlation between perceived voltage (mV) and the time from emergency to permanent pacing. Admission diagnosis has a significant positive impact on the time from emergency to permanent pacing. The change (increase) in time from emergency to permanent pacing was 1.137-fold when an additional condition was diagnosed on admission.

## Figures and Tables

**Figure 1:** Quadratic curve fitting (dot: observed value; line: quadratic curve fitting).

**Figure 2:** Ridge trace map.

**Table 1:** Basic information of 20 patients.

Features	Value
Sinus noD (*n*/%)	6 (30%)
Third-degree AVB (*n*/%)	15 (75%)
Advanced AVB (*n*/%)	1 (5%)
Ventricle tachycardia (*n*/%)	4 (20%)
Diagnostic diseases (species)	2∼4
Age (years)	64.55 ± 8.75
Gender (male/female)	16/6

**Table 2:** Summary of Poisson regression analysis results (*n* = 20).

Item	Regression coefficient	Standard error	*Z* value	*p* value	OR value	OR value, 95% CI
Cr	0.002	0.001	3.386	≤0.001	1.002	1.001∼1.003
BUN	−0.034	0.008	−4.573	≤0.001	0.966	0.952∼0.981
Intercept	4.822	0.045	106.316	≤0.001	124.157	113.598∼135.699

Dependent variable: HBG; McFadden's R formula: 0.100.

**Table 3:** Pearson correlation-detailed format.

		Ventricular tachycardia
Age	Correlation coefficient	−0.481^*∗*^
	*p* value	0.032

CK-MB	Correlation coefficient	0.458^*∗*^
	*p* value	0.042

CK	Correlation coefficient	0.523^*∗*^
	*p* value	0.018

^*∗*^*p* < 0.05.

**Table 4:** Pearson correlation-detailed format.

		Myocarditis
Age	Correlation coefficient	−0.669^*∗*^
	*p* value	≤0.001

CTnI	Correlation coefficient	0.838^*∗*^
	*p* value	≤0.001

^*∗*^*p* < 0.01.

**Table 5:** Summary of 5 Poisson regression analysis results (*n* = 19).

Item	Regression coefficient	Standard error	*Z* value	*p* value	OR value	OR value, 95% CI
AST	0.014	0.003	4.093	≤0.001	1.014	1.007∼1.020
ALT	0.004	0.001	3.506	≤0.001	1.004	1.002∼1.006
MYO	−0.003	0.001	−1.944	0.052	0.997	0.995∼1.000
CTnI	−0.553	0.215	−2.566	0.010	0.575	0.377∼0.878
Intercept	0.101	0.233	0.435	0.663	1.107	0.701∼1.747

Dependent variable: DDI; McFadden's R formula: 0.737.

**Table 6:** Summary table of curve regression coefficients.

	Nonstandardized coefficient		Normalization coefficient	*t*	*p*
	*B*	Standard error	Beta		
Constant	−193.880	99.964	—	−1.940	0.069
ALB	15.018	5.742	4.072	2.615	0.018^*∗*^
ALB'	−0.175	0.081	−3.381	−2.172	0.044^*∗*^

^*∗*^*p* < 0.05. Dependent variable: HBG.

**Table 7:** Summary of 7 Poisson regression analysis results (*n* = 19).

Item	Regression coefficient	Standard error	*Z* value	*p* value	OR value	OR value, 95% CI
Pro-BNP	−0.000	0.000	−6.033	≤0.001	1.000	1.000∼1.000
MYO	−0.000	0.000	−3.917	≤0.001	1.000	1.000∼1.000
ALB	0.027	0.004	6.991	≤0.001	1.028	1.020∼1.036
TBIL	0.004	0.000	11.708	≤0.001	1.004	1.003∼1.004
Intercept	4.152	0.171	24.318	≤0.001	63.582	45.498∼88.854

Dependent variable: PLT; McFadden's R formula: 0.603.

**Table 8:** Results of stepwise regression analysis (*n* = 19).

	Nonstandardized coefficient		Normalization coefficient	*t*	*p*	VIF	*R* ^*2*^	Adjust *R*	*F*
	*B*	Standard error	Beta						
Constant	26.524	1.554	—	17.072	≤0.001	—	0.516	0.488	*F* (1,17) = 18.150, *p* < 0.001
ALT	0.024	0.006	0.719	4.260	≤0.001	1.000			

Dependent variable: APTT, D-W value: 2.249.

**Table 9:** PLS regression: regression coefficients of the relationship between dependent variable *Y* and independent variable *X*.

	RBC	WBC	RBC (standardized)	WBC (standardized)
Constant	0.366	−5.934	0.000	0.000
BUN	−0.022	0.320	−0.126	0.300
AST	0.001	0.035	0.218	0.833
ALT	−0.002	0.000	−0.602	0.005
ALB	0.093	0.261	0.678	0.310
MYO	0.000	-0.001	0.011	−0.110
CTnI	0.262	0.301	0.424	0.079

**Table 10:** Results of stepwise regression analysis (*n* = 19).

	Non-standardized coefficient		Normalization coefficient	*T*	*p*	VIF	*R* ^*2*^	Adjust r	*F*
	*B*	Standard error	Beta						
Constant	0.906	0.021	—	43.730	≤0.001^*∗*^	—	0.592	0.568	*F* (1,17) = 24.625, *p* < 0.001
CK	0.000	0.000	0.769	4.962	≤0.001^*∗*^	1.000			

Dependent variable: INR, D-W value: 1.733, ^*∗*^*p* < 0.01.

**Table 11:** Adjustment effect analysis results-simplified format.

	Model 1	Model 2	Model 3
Constant	56.750^*∗∗*^(25.957)	56.750^*∗∗*^(26.908)	56.531^*∗∗*^(22.988)
Sinus node dysfunction	−10.833^*∗*^(−2.271)	−6.863 (−1.299)	−6.949 (−1.273)
Ventricular tachycardia	—	−9.265 (−1.531)	−10.038 (−1.348)
Sinus node dysfunction*∗*ventricular tachycardia	—	—	2.436 (0.190)
Sample size	20	20	20
*R* ^*2*^	0.223	0.317	0.318
Adjust r	0.179	0.236	0.191
variance ratio	*F* (1,18) = 5.156, *p*=0.036	*F* (2,17) = 3.942, *p*=0.039	*F* (3,16) = 2.491, *p*=0.097
△*R*^2^	0.223	0.094	0.002
△*F* value	*F* (1,18) = 5.156, *p*=0.036	*F* (1,17) = 2.343, *p*=0.144	*F* (1,16) = 0.036, *p*=0.852

Dependent variable: pacing frequency (times/min), ^*∗*^*p* < 0.05*t* value in parentheses.

**Table 12:** Adjustment effect analysis results-simplified format.

	Model 1	Model 2	Model 3
Constant	56.750 (26.408)	56.750 (26.908)	56.531 (22.988)
Ventricular tachycardia	−13.125^*∗*^(−2.443)	−9.265 (−1.531)	−10.038 (−1.348)
Sinus node dysfunction	—	−6.863 (−1.299)	−6.949 (−1.273)
Ventricular tachycardia*∗*sinus node dysfunction	—	—	2.436 (0.190)
Sample size	20	20	20
*R* ^*2*^	0.249	0.317	0.318
Adjust *R*	0.207	0.236	0.191
Variance ratio	*F* (1,18) = 5.968, *p*=0.025	*F* (2,17) = 3.942, *p*=0.039	*F* (3,16) = 2.491, *p*=0.097
△*R*^2^	0.249	0.068	0.002
△*F* value	*F* (1,18) = 5.968, *p*=0.025	*F* (1,17) = 1.687, *p*=0.211	*F* (1,16) = 0.036, *p*=0.852

Dependent variable: pacing frequency (times/min). ^*∗*^*p* < 0.05; *t* value in parentheses.

**Table 13:** Chi-square test analysis results.

Subject	Name	Sinus node dysfunction (%)		Total	*χ* ^2^	*p*
		0.0	1.0			
Third degree	0.0	1 (7.14)	3 (50.00)	4 (20.00)	4.580	0.032^*∗*^
Atrioventricular block	1.0	13 (92.86)	3 (50.00)	16 (80.00)		
Total	—	14	Six	20		

^*∗*^*p* < 0.05.

**Table 14:** Discriminant analysis: prediction accuracy of the training set.

Forecast category	Sample size	Accuracy (%)	Recall rate(%)	*F*1 score (%)
Category 1 (right subclavian)	3	0.00	0.00	0.00
Category 2 (within the right neck)	14	77.78	100.00	87.50
Class 3 (expensive to vein)	1	0.00	0.00	0.00
Summary	18	60.49	77.78	68.06

**Table 15:** Pearson correlation: detailed format.

		Perceived voltage (mV)	Pacing current (mA)
Emergency to permanent pacing time	Correlation coefficient	0.746^*∗*^	−0.470
	*p* value	0.013^*∗*^	0.170

Pacing threshold current (mA)	Correlation coefficient	−0.097	0.719
	*p* value	0.722	0.002^*∗∗*^

^*∗*^*p* < 0.05 and ^*∗∗*^*p* < 0.01.

**Table 16:** Summary of negative binomial regression analysis results (*n* = 10).

Item	Regression coefficient	Standard error	*Z* value	*p* value	OR value	OR value, 95% CI
Intercept	2.373	0.554	4.286	≤0.001	10.725	3.624∼31.739
Admission diagnosis	0.128	0.053	2.401	0.016	1.137	1.024∼1.262

Dependent variable: time from emergency to permanent pacing; McFadden's R formula: 0.017.

## Data Availability

The data used to support the findings of this study are included within the article and the supplementary information file.

## Supplementary Materials

Supplementary Materials Raw data for the SPSS analysis.
